The article "Efficiency Evaluation and Influencing Factors Analysis of Logistics Industry based on Multiobjective Intelligent Computing" was published in 2022. Journal: Comput Intell Neurosci.

# Efficiency Evaluation and Influencing Factors Analysis of Logistics Industry based on Multiobjective Intelligent Computing

**DOI:** 10.1155/2022/3098160

**Published:** 2022-08-23

**Authors:** Tingyan Zhou, Wenxing Li

**Affiliations:** School of Economics and Management, Beijing Jiaotong University, Beijing 100044, China

## Abstract

In logistics industry of 12 provinces along China's new western land-sea corridor from 2010 to 2019, this research employed three-stage SBM model that considers undesirable output to measure logistics industrial efficiency and the panel Tobit model to investigate variables impacting logistics efficiency. The study found that after controlling for environmental variables and statistical noise, the logistics industrial efficiency in China's new western land-sea corridor has improved, and the logistics sector efficiency of each province has spatial variability. Generally speaking, the south part goes up and the north part goes down; industrial structure, logistics transportation intensity, and economic development have a favorable influence on logistics sector efficiency. The urbanization rate, government support level, level of infrastructure, and degree of openness all have a negative influence on efficiency. Finally, relevant policy considerations such as logistics transport intensity, pure technical efficiency, scale efficiency, and external environment are proposed.

## 1. Introduction

From the mid-1990s to the present, as the economy develops, the logistics industry has developed rapidly. Logistics is an important strategic sector whose development is inseparable from the dynamics of other businesses. Despite China's logistics industry has developed rapidly, due to the continuous improvement of distribution capabilities, the proportion of total social logistics costs as a percentage of GDP has dropped from 18.0% in 1991 to 14.6% in 2017, the proportion remains significantly higher than in industrialized nations like Europe and the United States. The current situation is still a real problem for China's trade [1]. Most earlier studies on the relationship between logistics and economic returns produced biased results regardless of social and environmental concerns. However, the spatial temporal variations in China logistics efficiency are examined with undesired outcomes as well as the impact of other external factors, and the results show that the China's logistics is less efficient but will only improve over time [2].

The growth of the logistics industry of China's new western land-sea corridor will benefit the economy of western China and its surrounding countries, and the new western land-sea corridor may have fostered trade partnerships with other countries, boosting regional growth in western China and Southeast Asia [3]. Therefore, following a comprehensive assessment by a multisector computer model, this paper aims to evaluate system efficiency of the sustainable logistics industry based on combining inputs and desired and undesired outputs.

## 2. Literature Review

In regional logistics industry efficiency measurement methods, Data Envelope Analysis (DEA) has become the main method, which does not require to define certain production functions and processmeasurement data,norspecify the weights of the input-output indicators. Markovits-Somogyi and Bokor used the new DEA-PC method (pairwise comparison) to assess logistics efficiency in 29 European nations, and the results were analyzed by using Logistics Performance Index (LPI) [4]. Zahran et al. evaluated the efficiency of port taxation by using DEA and assessed their income generation mechanisms in terms of efficiency [5]. Lei et al. used the DEA-Malmquist approach to conduct an empirical research of the technical growth of 49 Chinese listed logistics enterprises from 2008 to 2017 [6]. Fried et al. proposed a three-stage DEA to reduce the impact of environment and statistical noise on decision-making units, with the positive objective of reflecting efficiency measurement result [7]. Qin used a three-stage DEA to quantify logistics efficiency in the 9 + 2 urban agglomeration of Guangdong, Hong Kong, and Macao from 2012 to 2018 and concluded that the impact of logistics sector fixed asset investment and the transportation network density on efficiency is extremely important [8].

In order to overcome the bias caused by the radial DEA, slack based measure (SBM) is presented, which considers not only slack variables but also desirable and undesirable outputs to improve efficiency measurement accuracy [9]. Wang and Liu used panel data from the Yangtze River Economic Zone logistics industry between 2005 and 2014 to quantify logistics sector efficiency with the Super-SBM accounting for undesirable output, and the results indicate that measuring logistics efficiency with undesirable output is close to the real distribution process [10]. Feng et al. used panel data of 17 Chinese port listed companies between 2010 and 2015, an empirical analysis is conducted with the SBM model, and conclusions were drawn on their overall operational efficiency [11]. Liu and Sun used the panel data from China's logistics sector between 2004 and 2014 to calculate the Super-SBM and Malmquist models with undesired output and concluded that the total factor productivity with undesired output is more realistic [12]. Ma et al. utilized a three-stage SBM to examine the logistics sector efficiency in Northeast China and six provinces in the “Yangtze River Delta” area from 2011 to 2015, which revealed that the logistics industry's technological efficiency and scale efficiency are higher in the “Yangtze River Delta” area than in the Northeast, and the small size of the logistics industry in the Northeast causes poor efficiency [13].

Some researchers have conducted relevant studies on the elements impacting logistics sector efficiency, and the research methods are mainly divided into three categories: (1) combine DEA and Tobit models to examine specific aspects of logistics efficiency. Zhou et al. analyzed Chinese 3PL enterprises efficiency using DEA and used multiple regression analysis to investigate the factors influencing 3PL efficiency [14]. Wang et al. analyzed China's road logistics efficiency and the elements that influence it and found that the central region has the highest road logistics efficiency and the western region has the lowest, but some western provinces have higher road logistics efficiency, and the level of regional informatization and road logistics resource utilization have the greatest influence on China's road logistics efficiency [15]. Gong et al. examined the effectiveness of China's logistics sector in 2017 and concluded that while there are significant disparities in logistics efficiency among areas, the amount of regional economic growth has minimal impact on logistics efficiency [16]. (2) Combine three-stage DEA and Tobit model to assess various aspects affecting logistics efficiency. Wong et al. utilized three-stage DEA to examine the efficiency of 77 logistics companies in Singapore and Malaysia between 2012 and 2013, and the Tobit model to examine the elements that impact logistics efficiency [17]. Zhang et al. analyzed the logistics sector efficiency of 19 provinces in the Yangtze River Reserve from 2013 to 2017, concluding that scale efficiency is a key factor influencing total efficiency [18]. (3) Combine SBM and Tobit model to examine the specific aspects affecting influencing logistics efficiency. Tian et al. studied the efficiency and its influencing factors of 90 fresh produce e-commerce enterprises in China from 2016 to 2017 and found that the overall technical efficiency of fresh produce e-commerce enterprises was low, and there was a significant positive effect of IT talent share structure, relationship with partners and logistics infrastructure level on the technical efficiency of fresh produce e-commerce enterprises, while there was a significant negative effect of information technology level [19]. Cao and Deng conducted an empirical analysis on the Yangtze River Economic Zone's logistics efficiency between 2007 and 2016 and analyzed the factors affecting logistics efficiency [20].

Therefore, previous research mostly focuses on the radial DEA or nonradial SBM for assessing the efficiency of logistics industry, without taking into account the influence of environment and statistical noise. Although the three-stage DEA reduces the influence of environmental factors and statistical noise, it ignores undesirable output and cannot guarantee the objectivity of efficiency measurement results. In addition, few studies have been conducted to systematically assess the logistics sector efficiency in China's new western land-sea corridor as the research topic. On this basis, this paper is extended as follows: (1) in the research method, considering the undesirable results, a three-stage SBM model is developed to calculate the logistics sector efficiency, and a panel Tobit model can be used to discuss the main influences elements on logistics sector efficiency. (2) In the research content, from 2010 to 2019, the panel data of logistics industry input-output indicators from 7 provinces, 4 autonomous regions, 1 municipality (henceforth referred to as 12 provinces) along China's new western land-sea corridor are selected for empirical analysis to identify the important influencing factors.

## 3. Research Design

### 3.1. Measure Model

#### 3.1.1. Three-Stage SBM Model

The first stage: slack-based measure (SBM) considering undesirable output.

Suppose there are *n* decision making units (DMU), each unit has *x* input indicators, *y*^*g*^ desirable output indicators, and *y*^*b*^ undesirable output indicators, assuming matrices *X*=[*x*_1_,…, *x*_*n*_] ∈ *R*^*m*×*n*^, *Y*^*g*^=[*y*_1_^*g*^,…, *y*_*n*_^*g*^] ∈ *R*^*s*_1_×*n*^, *Y*^*b*^=[*y*_1_^*b*^,…, *y*_*n*_^*b*^] ∈ *R*^*s*_2_×*n*^, and *X*>0, y^*g*^>0 and y^*b*^>0. The equation is as follows:

(1) $$\begin{array}{c} \rho =\text{min}\frac{1-1/m\sum_{i=1}^{m}s_{i}^{-}/x_{i0}}{1+1/s_{1}+s_{2}\left(\sum_{r=1}^{s_{1}}s_{r}^{g}/y_{r0}^{g}+\sum_{r=1}^{s_{2}}s_{r}^{b}/y_{r0}^{b}\right)}\\ \text{subject to}\left\{\begin{array}{c} x_{0}=X\lambda +s^{-}\\ y_{0}^{g}=Y^{g}\lambda -s^{g}\\ y_{0}^{b}=Y^{b}\lambda +s^{b}\\ s^{-}\geq 0,s^{g}\geq 0,s^{b}\geq 0,\lambda \geq 0. \end{array}\right. \end{array}$$

In the above formula: *ρ* is the efficiency, and 0 ≤ *ρ* ≤ 1; *s*^−^ ∈ *R*^*m*^ is the input slack variable; *s*^*g*^ ∈ *R*^*s*_1_^ is the desirable output slack variable; *s*^*g*^ ∈ *R*^*s*_2_^ is the undesirable output slack variable; *λ* ∈ *R*^*n*^ is the weight variable.

The second stage: stochastic frontier analysis(SFA)

The equation is measured as follows by using SFA:

(2) $$\begin{array}{c} s_{ni}=f^{n}\left(z_{i};\beta^{n}\right)+v_{ni}+\mu_{ni}\text{,}n=1,\ldots ,N,i=1,\ldots ,I. \end{array}$$

Among them, *s*_*ni*_ is the slack variable of item *n* of the *i* DMU's input; *f*^*n*^(*z*_*i*_; *β*^*n*^) is the influence of environmental variables on *s*_*ni*_; *z*_*i*_=(*z*_1*i*_, *z*_2*i*_,…, *z*_*ki*_) is the *k* environmental variables; *β*^*n*^ is the environmental variables coefficient; *v*_*ni*_ is the statistical noise; *μ*_*ni*_ is the managerial inefficiency.

Using the results of SFA to alter the input variables, all decision-making units are modified to the similar situations, the equation is as follows:

(3) $$\begin{array}{c} x_{ni}^{A}=x_{ni}+\left[\max\left(f\left(z_{i};{\hat{\beta }}^{n}\right)\right)-f\left(z_{i};{\hat{\beta }}^{n}\right)\right]+\left[\max\left({\hat{v}}_{ni}\right)-{\hat{v}}_{ni}\right]\text{,}n=1,\ldots ,N,i=1,\ldots ,I, \end{array}$$

where: *x*_*ni*_^*A*^ is the modified input variable, *x*_*ni*_ is the original input variable before modification. $\left[\max\left(f\left(z_{i};{\overset{⌢}{\beta }}^{n}\right)\right)-f\left(z_{i};{\overset{⌢}{\beta }}^{n}\right)\right]$ represents the adjustment for external environmental influences, and $\left[\max\left({\hat{v}}_{ni}\right)-{\hat{v}}_{ni}\right]$ represents the adjustment for statistical noise.

The third stage: after adjusting the input variables, carry out the SBM model analysis.

The adjusted input variable *x*_*ni*_^*A*^ obtained by formula (3) is used to replace the original input *x*_*ni*_ before adjustment, and the first-stage SBM is proposed again to assess the efficiency to obtain the real efficiency after excluding external environmental influences and statistical noise.

#### 3.1.2. Panel Tobit Model

Since the logistics sector efficiency assessed by the SBM in the third stage is in the [0,1] interval, which is not a normal distribution, it does not meet the assumption requirements of OLS for the normal distribution of the explained variables. Therefore, taking the logistics industry efficiency calculated by three-stage SBM model as the dependent variable, and various impacting factors on the logistics industry efficiency are used as independent variables, the equation is as follows:

(4) $$\begin{array}{c} y_{i}=\left\{\begin{array}{cc} y_{i}^{*}=X_{i}^{\prime }\beta +u_{i}, & y_{i}^{*}>0,\\ 0, & y_{i}^{*}\leq 0, \end{array}\right. \end{array}$$

where *y*_*i*_ is the efficiency; *y*_*i*_^*∗*^ is the potential dependent variable; *X*_*i*_′ is the independent variable; *β* is the coefficient; *u*_*i*_ is the statistical noise, *u*_*i*_ ~ (0, *σ*^2^)

Substitute the variables in Table 1 into formula (4) to construct a panel Tobit model:

(5) $$\begin{array}{c} y_{it}=\beta_{0}+\beta_{1}X1_{it}+\beta_{2}X2_{it}+\beta_{3}X3_{it}+\beta_{4}X4_{it}+\beta_{5}X5_{it}+\beta_{6}X6_{it}+\beta_{7}X7_{it}+u_{it}. \end{array}$$

Among them, *y*_*it*_ is the logistics industry efficiency; *β*_0_ is a constant term; *β*_1_ , *β*_2_,…, *β*_7_ is the regression coefficient; *u*_*it*_ is the statistical noise; *X*1_*it*_ is the urbanization rate; *X*2_*it*_ is the government support level; *X*3_*it*_ is the infrastructure level; *X*4_*it*_ is the industrial structure; *X*5_*it*_ is the degree of openness; *X*6_*it*_ is the logistics transportation intensity; *X*7_*it*_ is the economic development; *i* is the province; *t* is the time.

### 3.2. Indicator System

This paper selects indicators of the logistics industry and provides a suite of research indicator systems to assess the efficiency and influencing factors of the logistics sector in China's new western land-sea corridor, as indicated in Table 1.

#### 3.2.1. Input Indicator

Use labor force, capital, and energy as input indicators.

The work force is calculated by adding the total population employed in urban logistics units, urban private logistics firms, and individual logistics sector employees.

The capital stock formula is as follows:

(6) $$\begin{array}{c} K_{it}=K_{it-1}\times \left(1-\delta \right)+\frac{I_{it}}{P_{it}}. \end{array}$$

Among them, *K*_*it*_ and *K*_*it*−1_ represent the logistics industry's capital stock in *i* province in period *t* and *t* − 1, respectively; *K*_*i*0_ represents the logistics industry's capital stock in *i* province in its base period, divided by 10% of the fixed asset investment in 2010(2010 as the base period); *δ* represents the capital depreciation rate, which is taken as 9.6% [21]; *I*_*it*_ represents the fixed asset investment amount of *t* period of *i* province; *P*_*it*_ represents the price index of fixed asset investment of *t* period of *i* province.

The formula for calculating energy is as follows:

(7) $$\begin{array}{c} E=\sum_{i=1}^{11}\left(M_{i}\times P_{i}\right). \end{array}$$

Among them, *E* represents the total energy consumption of energy after the conversion to standard coal of various types of energy; *M*_*i*_ is the various types of energy involved in the logistics industry; *P*_*i*_ is the reference coefficient for the conversion to standard coal of the *i* energy.

#### 3.2.2. Output Indicator

Value added and carbon dioxide emissions are used as output indicators. Value added represents the desirable output and is processed by using the GDP deflator (2010 as the base period). Carbon dioxide emissions represent undesirable output and are computed as the sum of the logistics industry's energy consumption with the emission factors provided by IPCC 2006 Guidelines.

#### 3.2.3. Environmental Variables

Complex environmental factors affect the efficiency of the logistics industry, but they are independent of the logistics industry itself. Four indicators are selected as environmental variables: economic condition, computerization development level, industrial market structure, import and export. Considering the availability of relevant indicators and the requirements of indicator selection, GDP is selected as the surrogate variable for economic condition, the mobile phone users at the end of the year is selected as the surrogate variable for computerization development level, the amount of registered legal entities in the logistics sector is selected as the surrogate variable for industrial market structure, and total import and export is selected as the surrogate variable for import and export.

#### 3.2.4. Influencing Factors

Seven factors influencing logistics sector efficiency are selected: urbanization rate, government support level, infrastructure level, industrial structure, logistics transportation intensity, degree of openness, and economic development.

1. Urbanization rate (X1): with the development of spatial structure and economic structure, the strong agglomeration of industries and population in the urbanization process and the change in distribution cost of logistics industry will affect the agglomeration of logistics industry. This paper describes the urbanization rate in terms of the share of urban population to overall population in each province.
2. Government support level (X2): the government can improve logistics infrastructure by providing effective logistics development strategies and financial support. At the same time, ineffective government intervention has also delayed the improvement of logistics competitiveness to a certain extent. This article reflects the level of government support through the ratio of logistics industry fiscal expenditure to the general budget expenditure of each province.
3. Infrastructure level (X3): the construction of transportation infrastructure network can improve the service capacity of the logistics sector. The ratio of the sum of railroad mileage, inland waterway mileage, and road mileage of each province to the area of each province is chosen to reflect the degree of infrastructure in each province.
4. Industrial structure (X4): the service demand for logistics industry in the tertiary industry exceeds that in the secondary sector, and the logistics sector demand composition is constantly changing. This paper selects the proportion of tertiary sector added value to GDP in each province to represent the industrial structure.
5. Degree of openness (X5): the expansion of the degree of openness can improve the level of local logistics technology and management, which in turn affects the logistics industry efficiency. The ratio of total exports and imports to GDP in each province is selected to represent the level of openness.
6. Logistics transportation intensity (X6): this paper selects the ratio of the total logistics turnover to the GDP of each province to represent the logistics transportation intensity.
7. Economic development (X7): the development of regional economy can provide relevant supporting facilities, human resources, scientific and technological foundation for the logistics industry, which in turn effects the logistics sector efficiency. This study utilizes real GDP per capita to assess the economic progress of each province.

### 3.3. Data Analysis

This paper selects the transportation, warehousing, and postal industries of 12 provinces along China's new western land-sea corridor between 2010 and 2019 as the research object to study the logistics industry. Tibet is excluded from the research scope owing to lack of statistics data. All research data came from the National Bureau of Statistics' website and the China Energy Statistical Yearbook (see Table 2 for details).

The correlation test of input and output indicators of logistics industry was carried out by stata16, the correlation coefficients are positive and pass the test at 1% significance level, which indicates that the indicators are reasonably chosen.  Table 3 displays the results.

## 4. Three-Stage SBM Model Results and Analysis

### 4.1. The First Stage

Based on the input-oriented SBM, MaxDEA Pro8 is used to assess the logistics sector efficiency in China's new western land-sea corridor between 2010 and 2019, as shown in Table 4. Technological efficiency, pure technological efficiency, and scale efficiency have averages of 0.71, 0.84, and 0.85, respectively, all of which do not reach DEA effectiveness. By province, the logistics industry's uneven development is more prominent, and its efficiency level varies greatly. The top three logistics industry efficiency averages are Ningxia, Inner Mongolia, and Shaanxi, all above 0.9, close to the frontier of efficiency levels. The bottom three logistics industry efficiency averages are Hainan, Qinghai, and Sichuan, which are all below 0.6. Among them, the explanation for Sichuan and Qinghai's poor average technical efficiency is low scale efficiency, while the low technical efficiency in Hainan is due to the low pure technical efficiency. Only five provinces have an average technical efficiency of more than 0.71, namely Ningxia, Inner Mongolia, Shaanxi, Gansu, and Guizhou, most of which are located in the northern portion of the new western land-sea corridor.

### 4.2. The Second Stage

Based on the SFA, the explained variables are the input slack variables collected in the first stage, as well as four environmental elements, namely, GDP, the mobile phone users at the end of the year, the amount of registered legal entities in the logistics sector, and total import and export are used as explanatory variables, and the frontier4.1 is used to examine whether environmental factors have a considerable influence on input slack variables.  Table 5 displays the results.

From Table 5, it can be concluded that:

  Economic condition: the economic condition represented by GDP is negatively associated with all three slack factors and passes the significance test. It shows that improving economic conditions can minimize input redundancy of capital stock, employees, and energy consumption, and reasonable deploy of resources to increase the overall logistics business efficiency.
  Computerization development level: the level of computerization represented by the mobile phone users at the end of the year is positively correlated with the slack variables “fixed assets” and “energy consumption,” and negatively correlated with the slack variable “employees,” all of which pass the test at the 1% statistical significance. It demonstrates that an increase in phone users at year end can result in increase in input redundancy of capital stock and energy consumption, resulting in inefficient allocation of capital and energy, while reducing the redundancy of employee input and making the employee input more reasonable.
  Industrial market structure: the industrial market structure, represented by the amount of registered legal entities in the logistics sector, is positively correlated with the slack variable of energy consumption and negatively correlated with the slack variable of capital stock, both of which pass the test at the 1% significance level. There is no significant relationship with the slack variable of employees. This shows that the increase in the number of registered legal entities in the logistics sector may lead to inefficient energy consumption and more rational allocation of capital.
  Import and export: total imports and exports is positively correlated with the slack variable of employees and energy consumption, and they pass the 1% significance test. It indicates that increasing import and export can lead to redundancy of employees and energy consumption, resulting in unreasonable input of employees and inefficient use of energy in the logistics industry.

### 4.3. The Third Stage

The second stage's modified input variables and the first stage's initial outputs are fed to the SBM of the first stage for calculation and give the real logistics industry efficiency.  Table 6 displays the results.

The third-stage logistics industry efficiency in different provinces is shown in Figure 1:

By province, there are obvious disparities in the logistics sector efficiency before and after the adjustment of each province. Inner Mongolia and Shaanxi's logistics sector efficiency always remains at the forefront. The technical efficiency in Ningxia, Hainan, Qinghai, Gansu, and Guizhou declines, and the technical efficiency of Chongqing, Guangxi, Sichuan, Yunnan, and Xinjiang improves. This shows that the first-stage SBM does not consider the impact of environmental factors and statistical noise; it is responsible for underestimating the logistics sector efficiency in some provinces with better environment. The logistics sector efficiency in better-off provinces cannot objectively reflect the real level of logistics industry efficiency. Environmental variables in different provinces have different effects on the technical efficiency of the logistics industry. After controlling for environmental factors and statistical noise, the largest changes in technical efficiency rankings include Sichuan (up 6 places) and Ningxia (down 8 places); the largest changes in pure technical efficiency rankings include Hainan (up 4 places), Chongqing, Sichuan, and Guizhou (down 2 places); and the largest changes in scale efficiency rankings include Chongqing (up 6 places) and Ningxia (down 9 places). Among them, the technical efficiency improvement areas are Sichuan, Yunnan, Chongqing, Guangxi, Guizhou, Inner Mongolia, Shaanxi, and the pure technical efficiency areas are Hainan, Guangxi, Gansu, maintaining the original ranking of Inner Mongolia, Yunnan, Qinghai, Ningxia, and Xinjiang, and scale efficiency ranking changes in Chongqing, Sichuan, Guangxi, Inner Mongolia, and Yunnan were the provinces with the highest efficiency levels, and Qinghai maintains the original ranking. The average technical efficiency in Guangxi has adjusted from 0.656 to 0.904, mainly due to pure technological efficiency improvement. Chongqing's average technological efficiency has increased from 0.685 to 0.917, mainly due to the improvements in both pure technological efficiency and scale efficiency. Qinghai and Ningxia's technological efficiency have decreased from 0.544 to 0.961 before adjustment to 0.259 and 0.697 after adjustment, respectively. The pure technical efficiency of the two provinces has been at the production frontier, so the reduction in technical efficiency is mostly related to the reduction in scale efficiency. The phenomenon of high technical efficiency in the first stage is partly due to external environmental variables. Hainan, Guizhou, Gansu, and Xinjiang have improved their pure technological efficiency, while their scale efficiency has declined, leading to a slight drop in logistics industry efficiency, showing that external environmental variables have not significantly driven the logistics sector development. The average technical efficiency of 6 provinces of Inner Mongolia, Shaanxi, Chongqing, Guangxi, Yunnan, and Sichuan exceeds 0.734, most of which are located in the southern half of the new western land-sea corridor.

## 5. Analysis of Influencing Factors

Panel Tobit model regression is performed by Stata16, and the results are shown in Table 7.

1. The effect of urbanization rate: the urbanization rate has significantly negatively correlated with the logistics sector efficiency. If the proportion of urban population to the total population in each province increases by 1 unit, the efficiency of the logistics sector will decrease by 3.5985, which means that the logistics industry's efficiency cannot be significantly improved as the urban population grows. Although the provinces of the new western land-sea corridor are accelerating the process of new urbanization, it will take a long time to push the growth of regional large logistics hubs and intracity logistics systems.
2. The influence of government support level: the degree of government funding has no obvious negative impact on logistics business efficiency. If the share of fiscal expenditure on the logistics sector in the general budget expenditure of each province increases by 1 unit, the efficiency of the logistics sector will decrease by 0.4964, indicating that there is no positive relationship between the government's fiscal expenditure on logistics industry and logistics business efficiency. Despite significant investments in logistics infrastructure by local governments, the logistics business in various provinces remains unequal.
3. The impact of infrastructure level: the transportation infrastructure network has a considerable negative impact on the logistics sector efficiency. If the share of the length of transport lines to the national territory in each province increases by 1 unit, the logistics sector efficiency will decrease by 0.3267. It shows that the increase in infrastructure construction cannot considerably enhance logistics sector efficiency. The convenient transport infrastructure network can help the logistics sector more efficient, but the redundant construction of the transport infrastructure will waste logistics resources.
4. The effect of industrial structure: the impact of industrial structure on logistics sector efficiency is not significant. If the share of value added in the services sector to GDP in each province increases by 1 unit, the efficiency of logistics industry will increase by 0.5721. This suggests that the industrial structure will lead to an increase in the efficiency, but the impact is not prominent. The development of the service sector contributes to service innovation in the logistics sector, the continuous satisfaction of different logistics services needs, and the continuous optimization of the resource allocation.
5. The impact of the degree of openness: the degree of openness has a considerable adverse influence on the logistics sector efficiency. If the share of total import and export to GDP of each province increases by 1 unit, the logistics sector efficiency will decrease by 0.5664. The majority of new western land-sea corridor is located in China's interior and its openness to the outside world is not high, which affects the flow of production factors and leads to the decrease of logistics sector efficiency.
6. The impact of logistics transportation intensity: logistics transportation intensity has a strong positive influence on logistics sector efficiency, when the ratio of total logistics turnover to GDP in each province increases by 1 unit, logistics sector efficiency increases by 1.0097. It indicates that the growth of logistics sector along the new western land-sea corridor should increase the value added while decreasing energy consumption of logistics industry by improving transportation intensity.
7. The influence of economic development: the economic development of each province has a substantial positive impact on the logistics sector efficiency, when each province's GDP per capita increases by 1%, the logistics sector efficiency increases by 0.5113%, implying that economic development leads to the improvement of logistics efficiency. Provinces with high level of economic development have a stable industrial base and sound industrial structure, which in turn promote the improvement of logistics industry efficiency.

## 6. Conclusion and Suggestion

Based on the growth of the logistics sector in 12 provinces of China's new western land-sea corridor from 2010 to 2019, this paper has introduced a three-stage SBM model considering nonradial, nonoriented, and undesirable output to make quantitative analysis of logistics efficiency and analyzes the influencing factors of logistics efficiency by using panel Tobin model and gets the following conclusions:

First, there are spatial variability of the logistics industry efficiency among provinces. From 2010 to 2019, except for Inner Mongolia, where the logistics sector's adjusted efficiency was at the production frontier. The logistics sector's efficiency in other provinces was uneven. The adjusted logistics sector efficiency of Shaanxi and Chongqing remains stable, while the logistics sector efficiency of Qinghai, Xinjiang, and Hainan was weak.

Second, the influence of environmental variables on logistics sector efficiency is diverse. Economic condition, computerization development level, industrial market structure, and import and export have a significant influence on logistics sector efficiency. There seem to be significant differences in logistics sector efficiency before and after adjustment.

Third, the panel Tobit model regression results indicate that industrial structure, logistics transportation intensity and economic development have positive effects on logistics sector efficiency, while urbanization rate, government support, infrastructure level, and degree of openness have negative effects on logistics business efficiency. Urbanization rate, infrastructure level, degree of openness, logistics transportation intensity, and economic development have significant effects on logistics industry efficiency, while government support and industrial structure have little effects on logistics industry efficiency.

In light of the findings, the following proposals are made in this paper:

The first is to improve current logistics transportation intensity of China's new western land-sea corridor. Promote the development of multimodal transit and land-sea intermodal transportation by railroad, highway, and waterway; support inland transport to speed up the adjustment of the transport structure; and increase the proportion of railway and waterway cargo transportation to the total freight volume. Rail and river transport for bulk transport has significantly reduces the cost of transporting raw materials, freight, and port transportation promote and facilitates the development of railway container distribution centers through rail-sea combined transportation and international trains, and strengthen intracorridor and cross-corridor cooperation. Ensure the smooth flow of the Southbound international railway and sea transport; promote the development of ports; improve the service level; formulate practical customs policies; and improve the comfort of pass customs.

The second is to improve the pure technological efficiency and scale efficiency of the logistics sector in the new western land-sea corridor. Make full use of the opportunity of creating “new infrastructure”; implement digital and intelligent logistics systems; expand the scope of information exchange; and improve the capabilities of logistics enterprises. Establish intelligent logistics industrial park; combine logistics with production factor policies; and develop the scale and benefits of logistics industrial parks.

Third, create a good external environment for logistics development in China's new western land-sea corridor. Considering the heterogeneity among environmental variables in different provinces, the change of environmental variables leads to significant changes in logistics efficiency in different provinces. All provinces should combine their own advantages, take enterprises as the main body under the leadership of the state, plan and standardize logistics industry growth, formulate and improve the logistics sector strategy, and promote the growth and introduction of green technology.

## Figures and Tables

**Figure 1:** Third-stage logistics industry efficiency.

**Table 1:** Efficiency measurement and influencing factor index system of logistics industry.

Indicator type	Metric name	Metric definitions	Unit
Input	Labor force	People employed in urban units in the logistics industry	10,000 people
	Capital	Logistics industry total social fixed asset investment	100 million yuan
	Energy	Logistics industry energy consumption	10,000 tons of standard coal

Desirable output	Value added	Logistics industry value added	100 million yuan
Undesirable output	CO_2_ emissions	CO_2_ emissions from the logistics industry	10,000 tons
Environmental variables	Economic condition	Gross domestic product (GDP)	100 million yuan
	Computerization development level	The mobile phone users at the end of the year	10,000 households
	Industrial market structure	The amount of registered legal entities in the logistics sector	Piece
	Import and export	Total import and export	Billion dollars

Influencing factors	Urbanization rate	Urban population/total population	%
	Government support level	Financial expenditure of the logistics industry/fiscal general budget expenditure	%
	Infrastructure level	Length of transportation route/land area	km/km^2^
	Industrial structure	Added value of tertiary industry/GDP	%
	Degree of openness	Total import and export/GDP	%
	Logistics transportation intensity	Total turnover of the logistics industry/GDP	Tons of km/yuan
	Economic development	Real GDP per capita	Chinese yuan/person

**Table 2:** Descriptive statistics of the efficiency measurement and influencing factors.

Indicator type	Metric name	Sample size	Average value	Standard deviation	Minimum	Maximum
Input	Labor force (100 million yuan)	120	7893.05	5676.19	1188.36	29314.7
	Capital (10,000 people)	120	342.86	259.79	46.5	1175.5
	Energy (10,000 tons of standard coal)	120	728.79	391.62	110.77	1715.84

Desirable output	Value added (100 million yuan)	120	533.16	330.82	70.7	1473.1
Undesirable outputs	CO_2_ emissions (10,000 tons)	120	1793.21	958.19	285.35	4083.73
Environment elements	Economic condition (100 million yuan)	120	10829.42	8099.97	1144.2	43169.27
	Computerization development level (10,000 households)	120	2670.01	1800.94	290.3	9443.5
	Industrial market structure (piece)	120	5623.53	4161.65	471	19283
	Import and export (billion dollars)	120	241.01	235.78	5.45	984.01

Influencing factors	Urbanization rate (%)	120	0.5	0.07	0.34	0.67
	Government support level (%)	120	0.08	0.02	0.04	0.16
	Infrastructure level (km/km^2^)	120	0.62	0.46	0.09	2.20
	Industrial structure (%)	120	0.51	0.05	0.35	0.63
	Degree of openness (%)	120	0.12	0.09	0.01	0.44
	Logistics transportation intensity (tons km/yuan)	120	0.26	0.14	0.06	0.65
	Economic development (yuan/person)	120	35137.26	12264.26	12882.00	71333.96

**Table 3:** Pearson correlation analysis on input-output indicators.

Input-output indicators	Logistics industry total social fixed asset investment	People employed in urban units in the logistics industry	Logistics industry energy consumption
Logistics industry value added	0.873^*∗∗∗*^	0.815^*∗∗∗*^	0.874^*∗∗∗*^
CO_2_ emissions from the logistics industry	0.870^*∗∗∗*^	0.712^*∗∗∗*^	0.998^*∗∗∗*^

*Note.* ^*∗∗∗*^ means significant at the 1% level.

**Table 4:** First-stage logistics industry efficiency.

Province	Technical efficiency	Ranking	Pure technical efficiency	Ranking	Scale efficiency	Ranking
Inner Mongolia	0.913	2	1	1	0.913	3
Guangxi	0.656	7	0.752	9	0.879	8
Hainan	0.581	10	0.699	10	0.825	10
Chongqing	0.685	6	0.831	6	0.847	9
Sichuan	0.532	12	0.817	8	0.671	11
Guizhou	0.740	5	0.817	7	0.907	5
Yunnan	0.615	9	0.669	12	0.901	6
Shaanxi	0.855	3	0.956	4	0.899	7
Gansu	0.796	4	0.882	5	0.908	4
Qinghai	0.544	11	0.972	3	0.560	12
Ningxia	0.961	1	1	1	0.961	1
Xinjiang	0.645	8	0.688	11	0.931	2
Maximum	0.961		1		0.961	
Minimum	0.532		0.669		0.560	
Average	0.71		0.84		0.85	

*Note.* Provincial averages for technical efficiency, pure technical efficiency, and scale efficiency range from 2010 to 2019.

**Table 5:** SFA regression results in the second stage.

Variable	Slack variable in capital stock	Employee slack variable	Slack variable in energy consumption
Constant term	−550.08 (−1.58)	12.75 (0.9)	8.63 (0.5)
GDP	−12170.52^*∗∗∗*^(−15.18)	−421.26^*∗*^(−1.74)	−2824.5^*∗∗∗*^(−6.7)
The mobile phone users at the end of the year	78220.58^*∗∗∗*^(177.01)	−599.99^*∗∗∗*^(−2.74)	2161.98^*∗∗∗*^(5.13)
The amount of registered legal entities in the logistics sector	−1778.34^*∗∗∗*^(−4.29)	−415.43(−0.71)	3468.94^*∗∗∗*^(4.95)
Total import and export	296.32(0.34)	415.78^*∗∗∗*^(6.41)	231.79^*∗∗∗*^(3.01)
Sigma-squared	6601762.7^*∗∗∗*^(2627652.00)	13050.99^*∗∗∗*^(66.78)	36212.3^*∗∗∗*^(6556.07)
Gamma	0.53^*∗∗∗*^(7.65)	0.58^*∗∗∗*^(10.71)	0.73^*∗∗∗*^(20.83)
Log likelihood function	−1076.76	−717.98	−740.05
LR test of the one-sided error	34.03^*∗∗∗*^	31.77^*∗∗∗*^	57.28^*∗∗∗*^

*Note.* ^*∗*^, ^*∗∗*^, ^*∗∗∗*^ indicate significant at 10%, 5%, and 1%, respectively, with the *t*-value enclosed in brackets.

**Table 6:** Third-stage logistics industry efficiency.

Province	Technical efficiency	Ranking	Pure technical efficiency	Ranking	Scale efficiency	Ranking
Inner Mongolia	1	1	1	1	1	1
Guangxi	0.904	4	0.976	7	0.926	4
Hainan	0.401	11	0.979	6	0.409	11
Chongqing	0.917	3	0.961	8	0.953	3
Sichuan	0.792	6	0.931	10	0.860	6
Guizhou	0.704	7	0.955	9	0.738	7
Yunnan	0.795	5	0.899	12	0.886	5
Shaanxi	0.969	2	0.984	5	0.985	2
Gansu	0.701	8	0.989	4	0.708	9
Qinghai	0.259	12	0.997	3	0.259	12
Ningxia	0.697	9	1	1	0.697	10
Xinjiang	0.665	10	0.921	11	0.723	8
Maximum	1		1		1	
Minimum	0.259		0.899		0.259	
Average	0.734		0.966		0.762	

*Note.* Provincial averages for technical efficiency, pure technical efficiency, and scale efficiency range from 2010 to 2019.

**Table 7:** Regression results of influencing factors on logistics industry efficiency.

*y*_*it*_	Coef.	Std. Err.	z	*P* > *z*
Urbanization rate	−3.5985^*∗∗∗*^	1.121	−3.21	0.001
Government support level	−0.4964	0.588	−0.84	0.398
Infrastructure level	−0.3267^*∗*^	0.187	−1.75	0.081
Industrial structure	0.5721	0.467	1.23	0.22
Degree of openness	−0.5664^*∗*^	0.305	−1.86	0.063
Logistics transportation intensity	1.0097^*∗∗∗*^	0.192	5.25	0
Economic development (take logs)	0.5113^*∗∗∗*^	0.169	3.02	0.003
Constant term	−2.9876^*∗∗*^	1.247	−2.4	0.017
Log likelihood	34.2272			
Prob > chi2	0			

*Note.* ^*∗*^, ^*∗∗*^, ^*∗∗∗*^ indicate significant at 10%, 5%, and 1%, respectively.

## Data Availability

The experimental data used to support the findings of this study are available from the corresponding author upon request.
